The article "An EEG Classification-Based Method for Single-Trial N170 Latency Detection and Estimation" was published in 2022. Journal: Comput Math Methods Med.

# An EEG Classification-Based Method for Single-Trial N170 Latency Detection and Estimation

**DOI:** 10.1155/2022/6331956

**Published:** 2022-02-18

**Authors:** Siyuan Zang, Xiaojun Ding, Meihong Wu, Changle Zhou

**Affiliations:** Department of Artificial Intelligence, School of Informatics, Xiamen University, Xiamen 361005, China

## Abstract

Event-related potentials (ERPs) can reflect the high-level thinking activities of the brain. In ERP analysis, the superposition and averaging method is often used to estimate ERPs. However, the single-trial ERP estimation can provide researchers with more information on cognitive activities. In recent years, more and more researchers try to find an effective method to extract single-trial ERPs, because most of the existing methods have poor generalization ability or suffer from strong assumptions about the characteristics of ERPs, resulting in unsatisfactory results under the condition of a very low signal-to-noise ratio. In this paper, an EEG classification-based method for single-trial ERP detection and estimation was proposed. This study used a linear generated EEG model containing templates of ERP local descriptors which include amplitude and latency, and this model can avoid the invalid assumption about ERPs taken by other methods. The purpose of this method is not to recover the whole ERP waveform but to model the amplitude and latency of ERP components. This method afterwards examined the three machine learning models including logistic regression, neural network, and support vector machine in the EEG signal classification for ERP detection and selected the best performed MLPNN model for detection. To get the utmost out of information produced in the classification process, this study also used extra information to propose a new optimization model, with which outperformed detection results were obtained. Performance of the proposed method is evaluated on simulated N170 and real P50 data sets, and the results show that the model is more effective than the Woody filter and the SingleTrialEM algorithm. These results are also consistent with the conclusion of sensory gating, which demonstrated good generalization ability.

## 1. Introduction

Electroencephalography (EEG) is a record of an electrogram of the electrical potentials on the scalp generated by the neurons of the brain. Due to its advantages of high temporal resolution, relative noninvasiveness, and lower cost of equipment, it is widely used in research such as cognitive science, neuroscience, and neural engineering.

Event-related potentials (ERPs) are also a measurement of brain activities occurring in a brain structure. Differing from the EEG signals, ERPs can only be evoked a short time after the brain receives a stimulus or event [1]. The ERPs can be viewed as the EEG changes after the brain is exposed to cognitive, sensory, or motor events. Since the mid-1980s, researches on ERPs have attracted a lot of attention [2]. An ERP waveform in a single trial may contain more than one component, and these components are usually described by its most distinctive features, which are called amplitude and latency. Each of the component provides meaningful information to many research areas including neuroscience, cognitive science, and psychophysiological research. For example, the P300 ERP component has a positive amplitude and exists with a latency of roughly 250 ms to 500 ms after decision-making, while the N170 ERP component has a negative amplitude and occurs with a latency of roughly 130 ms to 200 ms after the processing of familiar objects, faces, or words [3].

The article "An EEG Classification-Based Method for Single-Trial N170 Latency Detection and Estimation" was published in 2022. Journal: Comput Math Methods Med.

The ERPs have small amplitudes compared with the outside noises, artifacts, and spontaneous EEG, so the SNR may reach a considerable low value and even be negative. In order to extract the ERP components in the EEG signals, a superposition and average (SA) method [4] is often applied. However, many researches have been proposed to demonstrate that the SA technique has two obvious drawbacks. First, the validation of the SA method relies on a basic assumption that spontaneous EEG signals are absolutely random and stable with the mean value of zero so that they will be eliminated by the SA method [5]. However, this assumption is only approximately correct [6, 7] and not valid all of the time. Second, SA methods also make an assumption that ERP components triggered by the same stimulus are identical across trials. However, the researches demonstrated that ERPs repeatedly provoked by the invariant stimulus may be significantly different across trials in some cases [8–10]. Hence, the process of SA does not follow the basic principles of averaging. Moreover, it also prevents researches from trial-to-trial analysis because in the process of averaging, many kinds of meaningful and important information in cognitive science [11] are eliminated together with the spontaneous EEG signals.

Since the SA method is not suitable for some of the studies on cognitive science, many researchers are dedicated to finding an alternative method where the ERP components can be extracted from a single-trial EEG. So far, various methods have been suggested for the single-trial ERP estimation. Generally, these methods fall into two categories. Methods that fall into the first category use a single channel to estimate ERPs from the single-trial EEG. In 1967, with the help of correlation-averaging techniques, Woody [12] proposed a simple adaptive filtering model. With this model, the latency of an ERP component can be estimated from a single-trial EEG. Tuan et al. [13] applied a more advanced maximum likelihood technique to give estimation on the latency of ERP on a single-trial basis. This method assumed that the shape of the waveform and the amplitude of the ERP component is invariant. The following studies modified this maximum likelihood framework where the variation of amplitude can also be detected and estimated [5, 14]. Wavelet analysis [15–17] was another popular solution to this problem. Other classic single-channel techniques involve residue iteration decomposition and subspace-regularized least square method [18, 19]. The above methods using only a single channel are still important. However, it is not always easy to choose the best channel in many researches for the lack of prior knowledge. If researchers need to estimate multiple ERP components with multiple origins, these single-channel methods cannot perform well.

The article "An EEG Classification-Based Method for Single-Trial N170 Latency Detection and Estimation" was published in 2022. Journal: Comput Math Methods Med.

With the development of modern high-density EEG devices, a lot of information can be recorded from multiple electrodes. Many recorded spatial information can be used to extract ERP waveforms in considerable low SNR conditions with noisy EEG signals. Therefore, a variety of ERP extraction methods using multiple channels has been proposed. The most commonly used methods falling into this category include PCA [20, 21], ICA [22, 23], and sparse decomposition [24]. Among these techniques, ICA is probably the most successful and widely used method for ERP analysis. Spatially constrained ICA (scICA) [25], functional source separation (FSS) [26], and ICA-with-reference (ICA-R) [27] were introduced as the extension of traditional ICA. Other novel methods have also been proposed to solve this problem. Ranjbar et al. [28, 29] applied an advanced spatiotemporal filtering method where the Gaussian-shaped kernels were used to represent the ERP template. Huang et al. [30] proposed an ERP extraction method based on compressed sensing.

Recently, with the advances in machine learning, ERP analysis based on mathematical models and machine learning algorithms has attracted a lot of attention. Many of these methods are not designed specifically for single-trial ERP estimation but for ERP detection, but they can still provide insights into our work. Tang et al. [31] proposed a more advanced channel selection model combined with random forest and genetic algorithm for ERP detection. In addition to the application of the traditional machine learning method, the deep learning architectures have also been employed in ERP analysis in recent years. For ERP detection tasks, the most popular deep learning architectures are DBN [32], SAE [33], and CNN [34]. Each of the architectures achieved state-of-the-art classification accuracy on EEG classification for ERP detection.

The article "An EEG Classification-Based Method for Single-Trial N170 Latency Detection and Estimation" was published in 2022. Journal: Comput Math Methods Med.

However, current single-trial ERP estimations are faced with several problems. First, some of these methods still applied the invalid assumptions used in SA, which will produce errors in the estimation results. Second, some methods were only applied to estimate a certain form of ERP (such as P300), thus leading to poor generalization ability. Third, results produced by most of these methods had large errors in a very low SNR condition (especially for the estimation of peak latency). In this paper, we proposed an EEG classification-based method for single-trial ERP detection and estimation to address these problems.

Our method was implemented by improving and modifying the framework proposed by Huang et al. [35]. This framework contains a logistic regression model and a novel SingleTrialEM algorithm taking the mathematical properties of the objective equation in the optimization model into account to address this problem. It is a novel machine learning-based method to extract ERP because it not only detects ERP components in EEG signals but also makes use of the property of the classifier to give estimation of its amplitude and latency. The experimental result demonstrated that this method has a good generalization ability on real data, and it also performs much better than the Woody filter as well as on simulated data. However, this method has two significant drawbacks. First, although the logistic regression model is easy to apply with only a few parameters to be determined for the EEG classification task, the linear classifier produced by this model may have an unsatisfactory performance in the very low SNR condition, and this model also lacks flexibility. Second, the objective equation in this optimization model lacks sufficient robustness. This leads to the results predicted by this method to deviate from their ground-truth values.

To overcome these shortcomings, we examined the application of an artificial neural network (ANN) in EEG classification for ERP detection and compared the results obtained from logistic regression and support vector machine (SVM) and chose ANN as the most appropriate model for ERP detection. The SingleTrialEM regards the ongoing data recorded by EEG systems with multiple electrodes on the scalp as a matrix, and this is very suitable for EEG classification; we retained these advantages in our model. In addition, we carefully tested the structure of the neural network and the training algorithm to acquire a high accuracy as well as avoid overfitting. Since the EEG classifier produced by the neural network is nonlinear in this ERP detection task, this neural network classification model is more suitable for this task than logistic regression [36], and it can acquire higher accuracy. Besides, to get the utmost out of information produced by ANN in the classifying process, we used extra information to build our optimization model and abandoned the invalid part of the objective equation applied by SingleTrialEM. This modification was also proposed in our previous work [37].

The article "An EEG Classification-Based Method for Single-Trial N170 Latency Detection and Estimation" was published in 2022. Journal: Comput Math Methods Med.

In our improved framework, the invalid assumptions about ERP are totally abandoned. Besides, since the estimation results are correlated with the previous training process, our framework for ERP estimation can be applied in many scenarios. Moreover, with our more advanced optimization model, the estimation results of amplitude and latency can achieve high accuracy even in the very low SNR condition.

## 2. Materials and Methods

### 2.1. Subjects and Data Recording

A standard benchmark dataset [38] was used to evaluate the method on the real resting state EEG data. This study involves 21 participants who are all undergraduates with normal hearing and sight from the Texas State University. The data were recorded in a dark room, and all subjects were required to keep relax and awake during the process of recording to make sure that all data recorded were spontaneous EEG containing less noise. 72 channels of raw EEG signals of 8 minutes with 4 minutes of eyes closed and 4 minutes of eyes open were recorded from each participant in a resting state. The sampling rate was initially set to 2048 Hz and downsampled to 256 Hz afterwards. The placement of electrodes referred to the 10-5 international standards. An EEG system following that standard is shown in Figure 1.

To conduct the experiment on real data, we randomly selected 8 participants in Xiamen University with normal hearing and sight (sex ratio = 1 : 1, age range = 19–25), and the subjects were required to do three cognitive tests in this experiment (see Section 3.3 for details). For each subject, 16 channels of EEG signals of 17 minutes with 2 minutes of adjustment and 15 minutes of the task period were recorded. The sampling rate was 128 Hz. The placement of electrodes referred to the 10-20 international standards. According to these standards, the distances between adjacent electrodes are different from the 10-5 international standards, and the number of electrodes are fewer. This leads to different methods of selecting electrodes in brain regions in the experiment.

### 2.2. EEG Preprocessing and Feature Extraction

The raw EEG data has a high-multidimensional and noisy nature; a noisy looking waveform of EEG makes it difficult to do further analysis. All EEG data need to be preprocessed. The following steps were applied:

- *Filtering*. Before epoching or artifact removal, filtering continuous EEG data is often recommended. In this process, line noise and video noise are removed. We used a finite impulse response (FIR) filter to high-pass filter the raw EEG data at 1 Hz
- *Rereferencing*. Linked mastoids (LM) were used for referencing
- *Epoch extraction*. In this process, the EEG data was split into many fixed-size trials. Each epoch needs to contain a whole ERP component with no overlap with others. For example, since the ERP components we simulated in this paper were all N170, the length of each epoch was set according to 200 ms. Baseline correction was applied to remove the possible shifts in the baseline. The time range for baseline calibration was set to −100 ms to 0 ms (0 ms is the time point where the stimulus occurs)
- *Artifact removal*. In this process, we removed bad channels and bad data with visual inspection and automated rejection. The procedure of automated rejection was applied by an EEGLAB [39] plugin named Clean-rawdata. The parameters were set by referring to the official EEGLAB tutorial. Then, the process of removing saccade-related electroocular (EOG) artifacts and blink was applied referring to Trujillo et al. [38]. This is also the process of feature extraction

After preprocessing, the EEG data is much more informative and interpretable. Part of the preprocessed EEG data is demonstrated in Figure 2.

The article "An EEG Classification-Based Method for Single-Trial N170 Latency Detection and Estimation" was published in 2022. Journal: Comput Math Methods Med.

### 2.3. EEG Classification Method

Before estimating single-trial ERPs in our following framework, a classifier needs to be trained first to determine whether an EEG signal contains ERP or not.

#### 2.3.1. Logistic Regression

Traditional logistic regression is a frequently used technique for the linear classification task and estimation of the probability of certain events [40]. This method has many advantages; for example, the possibility of classification is modeled directly and we do not have to assume data distribution in advance so that the problem caused by inaccurate assumption on data distribution is avoided; since logistic regression forces the output value to lie between 0 and 1, this method not only gives estimation on data classes but also predicts probability, which is very useful for some tasks using probability to assist decision-making. Besides, the objective equation solved by logistic regression is a differentiable convex function of any order, which has good mathematical properties. The dichotomous outcome event is related to this equation:

(1) $$\begin{array}{c} \ln\frac{p\left(y=1\;|\;X\right)}{p\left(y=0\;|\;X\right)}=w^{\text{T}}X+b, \end{array}$$

where *b* represents the intercept, *w* represents the coefficient vector related to the EEG data sample *X*, and *p*(*y* = 1 | *X*) and *p*(*y* = 0 | *X*) are the probability that the sample *X* falls into a certain class.

The article "An EEG Classification-Based Method for Single-Trial N170 Latency Detection and Estimation" was published in 2022. Journal: Comput Math Methods Med.

Obviously, this equation can be converted into two equations:

(2) $$\begin{array}{c} p\left(y=1\;|\;X\right)=\frac{e^{w^{T}X+b}}{1+e^{w^{T}X+b}},\\ p\left(y=0\;|\;X\right)=\frac{1}{1+e^{w^{T}X+b}}. \end{array}$$

Therefore, we can estimate *w* and *b* by the maximum likelihood method. Given the dataset {(*X*_*i*_, *y*_*i*_)}_*i*=1_^*m*^, we can finally list the maximum likelihood function as well as the objective function to be solved:

(3) $$\begin{array}{c} l\left(w,b\right)=\arg\underset{w,b}{\max}\overset{m}{\underset{i=1}{\sum }}\ln p\left(y_{i}\;|\;X_{i};w,b\right). \end{array}$$

Many numerical optimization algorithms including the gradient descent method and Newton method can be used to solve this objective equation at an acceptable time complexity.

#### 2.3.2. Artificial Neural Networks

Artificial neural networks are typical machine learning methods to develop nonlinear classifiers, which have been used in BCI research [41, 42]. They consist of many simple, interconnected processing units named neurons. When the neuron is activated, it will send messages to connected neurons so that the potential in these neurons is changed; if the potential of a neuron exceeds a “threshold,” it will be activated and then send messages to other neurons.

In this paper, we only talk about the multilayer perceptron neural network (MLPNN) which is able to tackle nonlinear separable problems. It is composed of an input layer, one or several hidden layers, and an output layer. Input layer neurons receive input from the outside world (the EEG signals in our experiment), hidden layer and output layer neurons further process signals, and output layer neurons give the output of the final results (the classification results). More generally, MLPNN is fully connected and has no cross-layer connection or same-layer connection.  Figure 3 shows a structure of a fully connected neural network with one hidden layer.

*w* denotes the connection weight, *v* denotes the input of the hidden layer, and *ϕ* denotes the activation function which processes the output of neurons.

Theoretically, an MLPNN with enough neurons and layers is able to approximate any continuous function as well as classify any number of classes. Although this makes MLPNN very flexible, we do not have any prior knowledge about the number of hidden layers and nodes; too few nodes will lead to only a linear classification of the task and too many nodes will lead to the problem of overfitting. Besides, the training process will become more and more time consuming with the increase of structural complexity. In the present study, we carefully select each MLPNN's structure by trial and error.

The article "An EEG Classification-Based Method for Single-Trial N170 Latency Detection and Estimation" was published in 2022. Journal: Comput Math Methods Med.

#### 2.3.3. Support Vector Machine

The support vector machine is also widely used in the EEG classification task [43]. It is specifically designed for the 2 class classification task. The goal of an SVM is to find a classification hyperplane which can not only identify classes but also maximize the margins. With the “kernel trick,” the EEG data is implicitly mapped to a higher dimensional feature space so that it is possible to develop nonlinear decision boundaries. The “soft margin” including an undetermined regularization parameter *C* is introduced to allow errors on some samples. Unlike ANN, SVM directly deals with the task of good generalization ability and is insensitive to overfitting because it has fewer parameters to be defined by hand compared to ANN. If the kernel function is not chosen properly, it can lead to poor performance.

The choice of the kernel function is very important when using the SVM method. In BCI research, the most frequently used kernel is the Gaussian kernel [44]:

(4) $$\begin{array}{c} \kappa \left(X_{i},X_{j}\right)=e^{-{\left\|X_{i}-X_{j}\right\|}^{2}/2\sigma^{2}}, \end{array}$$

where *σ* denotes the width of the Gaussian kernel, which should be defined by hand. In our paper, we also use this kernel function to test the performance of SVM on the EEG classification task.

### 2.4. Linear Generative EEG Model

A basic assumption can be made that the electrical activities recorded at each channel by an EEG device can be viewed as a linear combination of multiple neural potentials [45]. What is more, the local descriptors of an ERP waveform vary across trials. Besides, spontaneous EEG signals cannot be viewed as absolutely stationary processes with a mean value of zero. Therefore, the linear generative EEG model is modeled as follows:

(5) $$\begin{array}{c} E_{D\times T}=\overset{R}{\underset{r=1}{\sum }}\sigma_{r}\cdot s_{r}{\left(\tau_{r}\right)}^{T}+X_{D\times T}, \end{array}$$

where *E* represents the EEG in a single trial, *σ*_*r*_ represents the amplitudes of ERP component *r* in different epochs, *R* represents the number of ERP components, *s*_*r*_ represents the waveform of ERP components from a trial, and *X* represents the spontaneous EEG signals from each trial with *T* samples. Researches show that the waveforms of ERP components are monophasic in most cases [2, 45]. The ERP component can be modeled by a template represented by f(*τ*) in the temporal domain, where *τ* represents the latency of an ERP component, multiplied by an undetermined parameter amplitude *σ*_*r*_. With this model, the problem to be solved is greatly simplified without violating the “neuronal generator” assumption of EEG data. The invalid assumption about ERP taken by some of the other single-trial ERP estimation methods is abandoned in this model, which can greatly improve the performance of our task.

The article "An EEG Classification-Based Method for Single-Trial N170 Latency Detection and Estimation" was published in 2022. Journal: Comput Math Methods Med.

In our task, the matrix *E* is already known in the above model; estimating *σ*_*r*_ and *τ*_*r*_ according to Equation (5) are the only problems that remain to be solved. These two undetermined parameters keep changing across trials in the model, which conforms to the actual situation. With this linear generative EEG model, estimating single-trial ERP becomes possible. However, we have to estimate 144 ( = 72 × 2) parameters for each ERP component in this model since on each channel, there are 2 undetermined parameters. It is almost impossible for us to apply this model without encountering any computational problem.

It is true that the ERP components in different electrodes are different according to previous studies [46, 47]. However, these studies also pointed that EPRs recorded by the electrodes placed on the same brain region can be seen as identical. Based on this fact, we can simplify the linear generative EEG model by putting ERP recorded by electrodes in the same brain region *Ω* in a group and estimating them simultaneously. In this group, the amplitude and latency of each ERP component can be regarded as the same. Moreover, we can select the time range *T* prudently, where there will be only one ERP component to be estimated. With these two steps, the number of undetermined parameters is reduced to 2. This method finally becomes workable without any computational problem, and the principles of neurophysiology are exactly followed [35]. The simplified model can be denoted by this equation:

(6) $$\begin{array}{c} E_{d\times t}=\sigma \cdot s\left(\tau \right)+X_{d\times t},d\in \Omega ,t\in T, \end{array}$$

where *σ* is a single number and *s* represents a matrix including *τ* where all row vectors are the same.

### 2.5. Template of ERP Component

We modeled a template of an ERP component by referring to Huang et al. [35]. It assumes that the ERP waveform is monophasic when it is triggered by an external stimulus. The form of this template is denoted by

(7) $$\begin{array}{c} f\left(\tau \right)=\exp\left(-\frac{{\left(t-\tau \right)}^{2}}{2\theta^{2}}\right), \end{array}$$

where *θ* denotes the width of the waveform. It is a constant for a given ERP component. We can build the simulation data according to the linear generative EEG model with a process of adding spontaneous EEG to the above template multiplied by an amplitude to be set manually.

The article "An EEG Classification-Based Method for Single-Trial N170 Latency Detection and Estimation" was published in 2022. Journal: Comput Math Methods Med.

With the linear generative EEG model and this template of the ERP component, we can easily model the simulated EEG data by generating a linear superposition of preprocessed spontaneous EEG and simulated ERP component. Besides, the optimization model in the framework for estimating ERPs also contains these two techniques.  Figure 4 shows the simulated N170 ERP component with an amplitude of 15 *μ*V. Figures 5 and 6 show spontaneous EEG data and its corresponding EEG signals containing ERPs.

### 2.6. Framework for Estimating ERPs

In the present work, the framework proposed in Huang et al. [35] was adopted. But we modified the framework by replacing the logistic regression classifier with a nonlinear one. For this purpose, we carefully compared the performance of logistic regression, artificial neural network, and support vector machine on the ERP detection task. Besides, the optimization model was also improved. The framework for estimating ERPs is illustrated by a flow diagram in Figure 7.

When the subject is not exposed to an outside event, the recorded EEG signals contain only spontaneous EEG. We marked these vectors as positive in the dataset. In contrast, when the subject receives an internal or external stimulus, an ERP component will be triggered. Even if we cannot predict the exact latency of the ERP components in each trial evoked by the same stimulus because the latencies are not always the same, the time range of their latencies is completely predictable according to the type of stimulus. We marked vectors in this range as negative samples in the dataset.

Therefore, for each subject, we are able to build a training set containing two classes of EEG signals. A classifier *Z* could be produced by neural network on the training set. We use Δ (*E* (*t*), *Z*) to represent the distance between *E* (*t*) and the classifier *Z*. The distance is positively correlated with the probability of *E* (*t*) to be positive. Then, we can convert the estimation of ERPs into an optimization problem using Δ(*E* (*t*), *Z*), Equation (6) can be converted to

(8) $$\begin{array}{c} X_{d\times t}=E_{d\times t}-\sigma \cdot s,d\in \Omega ,t\in T. \end{array}$$

If the time is fixed at one point, this equation can be redescribed as follows:

(9) $$\begin{array}{c} X_{d}\left(t\right)=E_{d}\left(t\right)-\sigma \cdot s\left(t-\tau \right),d\in \Omega ,t\in T. \end{array}$$

The time point close to the latency is marked as *T*^−^; the time point away from the latency is marked as *T*^+^. The selection of the time point is based on the width parameter *θ* in the template of ERP component mentioned in Section 2.5. A previous study [35] assumed that when $\hat{\sigma },\hat{\tau }$ approximate to their real values, these situations will appear: (1) when *T* ∈ *T*^−^, which class *X*_*d*_(*t*) belongs to, is not obvious to identify, as a result, Δ (*E*_*d*_ (*t*), *Z*) are almost equal to zero; (2) when *T* ∈ *T*^+^, *X*_*d*_(*t*) and *E*_*d*_(*t*) are almost identical because the ERP signals are hard to detect in the meantime. According to these two assumptions, the optimization model including one objective equation together with the SingleTrialEM algorithm was proposed as follows:

(10) $$\begin{array}{c} \hat{\sigma },\hat{\tau }=\arg\underset{\sigma ,\tau }{\min}\left(\underset{t\in T^{+}}{\sum }{\left(X_{d}\left(t\right)-E_{d}\left(t\right)\right)}^{T}\cdot \left(X_{d}\left(t\right)-E_{d}\left(t\right)\right)+\underset{t\in T^{-}}{\sum }\Delta \left(X_{d}\;\left(t\right),Z\right)\right). \end{array}$$

A specially designed SingleTrialEM algorithm which makes use of the mathematical properties of this model can be applied to tackle the optimization problem.

The article "An EEG Classification-Based Method for Single-Trial N170 Latency Detection and Estimation" was published in 2022. Journal: Comput Math Methods Med.

However, the objective equation built in this optimization model has two major disadvantages. First, if the results produced by the classifier have considerable high accuracy, the assumption (1) becomes invalid because sample classes in that time range are not difficult to predict. The nonlinear classifier trained by the artificial neural network can easily predict that *X*_*d*_(*t*) are positive samples because the ERPs will be eliminated from *E*_*d*_(*t*) if $\hat{\sigma },\hat{\tau }$ approximate to their real value. Second, though in our opinion, assumption (2) is still correct, the front part of Equation (10) based on this assumption will give an inaccurate estimation on the $\hat{\sigma }$ value in the process of optimization. Therefore, we abandoned this assumption and designed more effective objective equations.

To propose a better optimization model, two more valid assumptions were taken by us: (3) when *T* ∈ *T*^−^, Δ(*X*_*d*_(*t*), *Z*) from Equation (10) approximates to *D*. Δ (*X*_*d*_(*t*), *Z*) represents the distance between *X*_*d*_(*t*) and classifier *Z*. *D* represents the mean value of the distance between all *E*_*d*_(*t*) and *Z* in time range *T*^+^. (4) When *T* ∈ *T*^−^, the sum of Δ (*E*_*d*_(*t*), *Z*) will be the smallest near the latency because in this time range, the ERP signals should be strongest, which mean the samples in this time range are very likely to be negative. Based on these two assumptions, a much improved optimization model is proposed in this paper. In the redesigned optimization model, the unknown parameters, *τ* and *σ*, are estimated step by step:

(11) $$\begin{array}{c} \hat{\tau }=\arg\underset{\tau }{\min}\;\left(\underset{t\in T^{-}}{\sum }\Delta \left(E_{d}\left(t\right),Z\right)\right). \end{array}$$

Because the temporal resolution of the EEG device is limited and the range of the latency is predictable, latency *τ* can be regarded as a discrete interval variable. We can use a simple round-robin algorithm to solve this Equation (11). After having done estimating $\hat{\tau }$ of the latency *τ*, we should continue to determine the parameter *σ*:

(12) $$\begin{array}{c} \hat{\sigma }=\arg\underset{\sigma }{\min}\left(\underset{t\in T^{-}}{\sum }{\left(\Delta \left(X_{d}\left(t\right),Z\right)-D\right)}^{2}\right). \end{array}$$

Equation (12) is harder to solve; we can no longer use a round-robin algorithm like before since *σ* is a continuous variable. A built-in function in MATLAB named fminbnd which is designed for optimization problem on single-variable function is able to give estimation of this parameter given a fixed interval at an acceptable time complexity.

The article "An EEG Classification-Based Method for Single-Trial N170 Latency Detection and Estimation" was published in 2022. Journal: Comput Math Methods Med.

## 3. Results and Discussion

### 3.1. Experiment on Performance of Different EEG Classification Methods

In this section, we only show the performance of multiple EEG classification methods including logistic regression, artificial neural networks, and support vector machine on simulated data because the results are similar on real data.

As is mentioned in Section 2.2, before we conduct any experiment, data epochs must be extracted according to the stimulus onset. In our experiment on simulated data, the raw EEG signals were split into multiple 200 ms segments. All the trials were regarded as spontaneous EEG data with a time span of 200 ms according to the simulated stimulus onset. After that, with the linear generative EEG model, we can build the simulated data by superposing EEG trials with multiple channels on the template of the ERP component. All the templates were generated according to Equation (7) mentioned previously. We generated a simulated ERP component. The width *θ* value was set to 8 according to the neurophysiology plausibility of N170; latency *τ* value was set to 170 ms; and amplitude *σ* value was set to 3, 6, 10, and 15 *μ*M for each template. Each amplitude is corresponding to a suitable value of SNR levels. The main purpose of this paper is to test the performance in a very SNR condition, so the corresponding amplitudes were set at relatively low values. The parameter setting was referred to Huang et al. [35]. For each subject, the simulation data were divided into four sets with different amplitude values. Since the EEG signal strength measurements are based on power, the calculation of the SNR level should follow the “20 log” rule [48]:

(13) $$\begin{array}{c} \text{SNR}=20\cdot \log\left(\frac{\delta_{s}}{\delta_{n}}\right). \end{array}$$

6 pairs of vectors from the range of 162 to 178 ms from each spontaneous EEG trial were selected, and the raw data was marked as positive; data containing simulated ERP components was marked as negative. So the ratio of positive and negative samples in the EEG dataset was 1 : 1.

The article "An EEG Classification-Based Method for Single-Trial N170 Latency Detection and Estimation" was published in 2022. Journal: Comput Math Methods Med.

We selected the four brain regions according to the study in Huang et al. in [35]. The above four EEG datasets were divided into 16. Therefore, for each EEG classification method, we trained 16 models.

A logistic regression model was built by using 70% of the EEG data samples to derive the regression equations. The rest of the samples was left aside for model testing. A built-in function in MATLAB named glmfit was applied to develop the model; this function returns a vector of coefficient estimates for the given data. The distribution was set to “binomial” and its corresponding link function was set to “logit”, as is mentioned in Section 2.3.

Before we build the MLPNN model, we have to determine the number of hidden layers as well as the neurons in each hidden layer. Since we do not have any prior knowledge about which structure is best for our study, for each training set, we have to select the appropriate structure by trial and error. The original dataset was split into a training set, validation set, and test set, and the division ratio is 7 : 1.5 : 1.5. To choose the best structure of MLPNN, the validation set was used to measure network accuracy and generalization ability; it was also used to stop training when generalization stops improving. The Levenberg-Marquardt algorithm was adopted as the training algorithm because it costs less time and we do not need to worry about the memory problems. With the help of the validation set, we can rapidly tune the parameters of the MLPNN model. After determining the best structure of MLPNN for an EEG dataset (roughly the number of neurons were negatively correlated with the SNR level), the accuracy of the correctly classified EEG data was tested on the test set.

The process of building the SVM model was quite similar to MLPNN; the dataset was also split into a training set, validation set, and test set with the same proportion. But we only have to tune 2 parameters: the width of the Gaussian kernel *σ* and the regularization parameter *C*, which is also known as the box constraint. A built-in function in MATLAB named fitcsvm was applied to develop the SVM model.

The article "An EEG Classification-Based Method for Single-Trial N170 Latency Detection and Estimation" was published in 2022. Journal: Comput Math Methods Med.

The performance of these three methods is shown in Table 1. The results are the average accuracy of all 21 subjects and are sorted by the correctly classified rate.

It is obvious from the results that all methods performed better in the high SNR condition. The MLPNN trained with the Levenberg-Marquardt algorithm was at the top owing to its ability to predict ERP cases at the highest accuracy compared to the logistic regression and support vector machine. The MLPNN was able to gain an average of accuracy of more than 70% in three brain regions in the very low SNR conditions (in that case, the amplitude of simulated ERP components is 3 *μ*V), but it only produced slightly better classification results in the highest SNR condition than logistic regression. Accidentally, the support vector machine model trained with the Gaussian kernel had the lowest accuracy in this experiment. The possible reason is that we did not provide enough features of data samples (the samples were all 4-dimensional vectors) in order not to violate the assumption of Equation (6). This led to the poor generalization ability on the test set.

### 3.2. Experiment on Simulated Data

Based on the experimental results mentioned in Section 3.1, we chose the MLPNN to train the classifiers.

Three subjects from all the participants were randomly chosen for demonstration. The results are shown in Tables 2, 3, and 4. For the Woody filter, we chose one channel to replace a brain region because it is a single-channel method. The means and standard deviations of the results are demonstrated as a performance measurement.

The estimation results of latencies demonstrate that the performances of the SingleTrialEM and our method are both significantly better than that of the Woody filter. Even in high SNR conditions, the results of latencies produced by the Woody filter still largely deviate from the target value. As for the SingleTrialEM, the given results are much better, but there still exists 6–7 ms error between the mean values of latencies and the ground-truth value. What is more, the performance of this method does not get better with increase of SNR. In contrast, the latency results produced by our method are much more accurate. They are very close to the real value, and the errors of the mean value are no larger than 4 ms in any SNR level. Besides, the standard deviations become significantly smaller with the increase of SNR. This indicates that our objective Equation (11) makes the utmost of properties of the nonlinear classifier produced by MLPNN. However, our method has a large standard deviation in the very low SNR condition. The possible reason is that the objective equation we designed to estimate latency is just a simple process of summing and comparing the values, which may lead to instability in our estimation results.

The article "An EEG Classification-Based Method for Single-Trial N170 Latency Detection and Estimation" was published in 2022. Journal: Comput Math Methods Med.

As for the estimation results of amplitude, it can be concluded that the SingleTrialEM obviously underrated the amplitude values. By contrast, the mean values of amplitudes produced by our improved Equation.(12) are accurate in all the groups with the amplitude of 6–15 *μ*V. The standard deviations also go down in the high SNR condition. To further verify that our method outperformed the SingleTrialEM algorithm, two representative trials of the comparison of estimation results on the simulated N170 ERP component with an amplitude of 15 *μ*V between these two methods are presented in Figure 8. It is obvious from the figure that the results produced by our method are very close to the real value while the ERP waveform extracted by the SingleTrialEM has a significant offset from the real N170 ERP component.

We also used logistic regression to train the classifiers, and the estimation results of our method were still better than the SingleTrialEM but with worse performance. This further proves that the improvement of the training method and the modification of the optimization model both take effect in the single-trial ERP estimation task.

In this experiment on the simulated data, four brain regions including the left frontal, right frontal, left parietal, and right parietal were chosen for the experiment, but the selection of the regions are not limited to those; it varies with the experimental settings. Although ERPs have relatively low spatial resolution, they do provide some spatial information which can be used to identify their cortical origins [47]. For the N170 analysis, the brain regions can be selected by referring to some researches on the N170 localization [49, 50].

### 3.3. Experiment on Real Data

In addition to simulated data, we further verified our method with real data based on sensory gating. It is a neural process of the human brain of filtering out redundant information, which prevents an overload of information in the brain [51]. There are many techniques for sensory gating measurement; one of them is called the paired-click paradigm. According to sensory gating, if a subject hears a pair of sounds in a short period of time, the amplitude of the P50 ERP component evoked by the second sound will decrease significantly because it is perceived by the brain as being redundant [52].

Based on this mechanism of sensory gating, we performed three experiments containing delayed-response tasks with various memory loads. In task 1, the participants were asked to stay relaxed. In task 2, an image of a face was randomly selected as objective stimuli to keep the subject in a low-load object working memory state. In task 3, subjects were in a high-memory load with 2 images of randomly selected faces as objective stimuli. The subjects were required to keep the faces in mind and choose the same ones by clicking on the screen in tasks 2 and 3. In each task, all subjects were exposed to two sequential sounds.

The article "An EEG Classification-Based Method for Single-Trial N170 Latency Detection and Estimation" was published in 2022. Journal: Comput Math Methods Med.

According to the previous studies, the amplitude of the P50 ERP component triggered by the second sound should be significantly smaller than that of the P50 ERP component triggered by the first sound in all the three tasks. In this experiment, our framework for estimating single-trial ERPs was applied to estimate the single-trial P50 ERP components. By judging whether the experimental results are consistent with the phenomenon of sensory gating, we can verify our method on real data.

Subjects 1–4 took part in tasks 1 and 2, and subjects 5–8 were tested in tasks 1 and 3. The length of each trial was set to 100 ms. Vectors in the range of 0–16 ms were selected as positive samples, while vectors in the range of 42–58 were selected as negative samples because the latency of P50 has the better chance to be located in this range.

The results are listed in Table 5. It is obvious that the means of amplitude of the P50 triggered by the first sound are significantly larger than ones triggered by the second sound in all the 3 tests with the *P* value less than 0.05. The results are fully consistent with sensory gating, which further verifies our method on real data.

## 4. Conclusions

This paper proposed an event-related potential detection and estimation framework based on the EEG classification method. The framework consists of a linear generative EEG model, an MLPNN EEG data classifier, and an optimization model. Experimental results on simulated data showed that this method achieved satisfactory results in brain regions with various signal-to-noise ratios, and the results on actual data further demonstrated and validated the proposed method. With our purposed method, the local descriptors of an ERP component can be estimated accurately in the very low SNR condition without adopting the commonly used but invalid assumption about ERPs. Our method also has good generalization ability in many different ERP estimation tasks.

In our future work, we will try to improve our work by solving three main problems: First, the process of determining the structure of an MLPNN network for each dataset is very time consuming. More prior knowledge needs to be learned to simplify this process. Second, we did not test the performance of a more advanced deep learning algorithm for EEG classification. Third, a more advanced optimization model needs to be proposed to stabilize the results because the estimation of latency has a high standard deviation in very low SNR conditions. We are eager to tackle these problems in our future work.

The article "An EEG Classification-Based Method for Single-Trial N170 Latency Detection and Estimation" was published in 2022. Journal: Comput Math Methods Med.

## Figures and Tables

**Figure 1:** 10-5 international standard system.

**Figure 2:** Preprocessed EEG data of a subject with 32 channels and 5 epochs.

**Figure 3:** MLPNN structure.

**Figure 4:** Simulated N170 ERP components with an amplitude of 15 *μ*V.

**Figure 5:** Spontaneous single-trial EEG data of a subject with 4 channels.

**Figure 6:** Corresponding single-trial EEG data containing simulated N170 ERP components with an amplitude of 15 *μ*V.

**Figure 7:** Flow diagram for estimating ERPs.

**Figure 8:** Comparison of estimation results between the SingleTrialEM algorithm and the proposed algorithm.

**Table 1:** The results of different EEG classification methods.

Region	Amplitude	SVM	LR	MLPNN
Left frontal	3	52.54%	59.96%	67.56%
	6	59.79%	68.69%	73.72%
	10	70.08%	78.95%	82.74%
	15	82.61%	87.49%	90.16%
Right frontal	3	52.24%	60.89%	72.48%
	6	58.72%	70.24%	74.15%
	10	69.35%	79.23%	82.54%
	15	83.67%	87.16%	90.69%
Left parietal	3	53.78%	61.01%	70.86%
	6	62.05%	70.86%	74.09%
	10	70.04%	79.48%	83.32%
	15	80.61%	87.46%	90.41%
Right parietal	3	52.72%	58.92%	70.57%
	6	57.85%	67.48%	71.55%
	10	67.60%	76.16%	80.45%
	15	77.81%	84.66%	88.15%

**Table 2:** The results of simulation experiment on subject 1.

Region	Amplitude	SNR	Woody filter	SingleTrialEM		Ours	
				Amplitude	Latency	Amplitude	Latency
Left frontal	3	-31	103 ± 60	0.6 ± 0.7	177 ± 1	2.9 ± 1.7	171 ± 7
	6	-18	120 ± 60	2.5 ± 1.7	177 ± 2	5.9 ± 2.2	171 ± 6
	10	-7	142 ± 51	5.7 ± 2.5	177 ± 2	10.1 ± 2.2	171 ± 5
	15	1	163 ± 28	9.6 ± 3.0	177 ± 2	15.4 ± 2.2	171 ± 3
Right frontal	3	-31	103 ± 60	0.5 ± 0.7	177 ± 1	3.0 ± 1.6	171 ± 7
	6	-17	123 ± 59	2.4 ± 1.7	177 ± 2	6.3 ± 2.2	171 ± 6
	10	-7	142 ± 50	5.5 ± 2.6	177 ± 2	10.3 ± 2.3	171 ± 4
	15	2	160 ± 34	9.3 ± 3.0	177 ± 2	15.3 ± 2.3	171 ± 3
Left parietal	3	-30	98 ± 58	0.1 ± 0.7	177 ± 2	2.8 ± 1.7	168 ± 7
	6	-16	118 ± 58	1.4 ± 0.7	177 ± 2	5.6 ± 2.0	168 ± 6
	10	-6	145 ± 45	4.1 ± 2.4	177 ± 3	9.4 ± 2.2	168 ± 5
	15	2	164 ± 22	7.8 ± 2.5	177 ± 3	14.4 ± 2.3	169 ± 3
Right parietal	3	-35	100 ± 58	0.1 ± 0.6	177 ± 1	2.8 ± 1.7	170 ± 7
	6	-21	115 ± 57	1.1 ± 1.6	177 ± 2	5.6 ± 2.0	168 ± 7
	10	-11	133 ± 50	3.5 ± 2.6	177 ± 2	9.4 ± 2.2	168 ± 6
	15	-3	149 ± 38	6.9 ± 3.2	177 ± 2	14.4 ± 2.3	169 ± 4

**Table 3:** The results of simulation experiment on subject 2.

Region	Amplitude	SNR	Woody filter	SingleTrialEM		Ours	
				Amplitude	Latency	Amplitude	Latency
Left frontal	3	-32	76 ± 48	0.8 ± 0.9	177 ± 1	4.1 ± 2.3	174 ± 7
	6	-19	89 ± 56	3.0 ± 2.1	177 ± 1	6.3 ± 2.3	173 ± 6
	10	-8	137 ± 56	6.4 ± 3.0	177 ± 2	10.3 ± 2.3	172 ± 5
	15	0	158 ± 36	10.2 ± 3.5	177 ± 2	15.1 ± 2.3	172 ± 4
Right frontal	3	-31	103 ± 61	1.1 ± 0.9	177 ± 1	3.3 ± 1.7	173 ± 7
	6	-17	129 ± 58	3.8 ± 2.1	177 ± 1	6.5 ± 2.2	173 ± 5
	10	-7	151 ± 44	7.4 ± 2.8	177 ± 2	10.7 ± 2.2	172 ± 4
	15	1	163 ± 25	11.1 ± 3.2	177 ± 1	15.8 ± 2.3	172 ± 3
Left parietal	3	-32	79 ± 54	0.3 ± 0.9	177 ± 2	2.8 ± 1.7	168 ± 7
	6	-18	103 ± 59	1.8 ± 2.1	177 ± 3	5.9 ± 2.2	168 ± 6
	10	-8	142 ± 49	4.7 ± 3.0	176 ± 3	10.1 ± 2.4	168 ± 5
	15	1	157 ± 29	8.3 ± 3.3	177 ± 3	14.7 ± 2.3	169 ± 4
Right parietal	3	-34	103 ± 53	0.2 ± 0.7	177 ± 1	3.1 ± 1.6	167 ± 7
	6	-20	117 ± 52	1.4 ± 1.8	177 ± 2	5.8 ± 2.2	167 ± 6
	10	-10	131 ± 47	4.0 ± 2.8	177 ± 2	10.2 ± 2.4	168 ± 5
	15	-1	149 ± 37	7.5 ± 3.5	177 ± 2	15.2 ± 2.4	168 ± 4

The article "An EEG Classification-Based Method for Single-Trial N170 Latency Detection and Estimation" was published in 2022. Journal: Comput Math Methods Med.

**Table 4:** The results of simulation experiment on subject 3.

Region	Amplitude	SNR	Woody filter	SingleTrialEM		Ours	
				Amplitude	Latency	Amplitude	Latency
Left frontal	3	-32	100 ± 56	0.4 ± 0.6	177 ± 2	2.8 ± 1.7	171 ± 7
	6	-18	111 ± 57	1.8 ± 1.6	177 ± 2	5.9 ± 2.2	171 ± 6
	10	-7	134 ± 54	4.7 ± 2.3	177 ± 2	9.7 ± 2.4	170 ± 5
	15	1	155 ± 38	8.4 ± 2.8	177 ± 2	14.8 ± 2.3	170 ± 3
Right frontal	3	-31	112 ± 58	0.3 ± 0.5	177 ± 1	3.2 ± 1.7	170 ± 7
	6	-18	123 ± 58	1.7 ± 1.5	177 ± 2	6.1 ± 2.2	170 ± 6
	10	-7	147 ± 47	4.4 ± 2.3	177 ± 2	10.2 ± 2.4	170 ± 5
	15	1	160 ± 34	8.0 ± 2.8	177 ± 2	15.1 ± 2.5	170 ± 3
Left parietal	3	-31	86 ± 54	0.2 ± 0.7	177 ± 1	3.2 ± 1.7	170 ± 7
	6	-17	99 ± 59	1.5 ± 1.8	177 ± 2	6.1 ± 2.2	170 ± 6
	10	-7	131 ± 56	4.3 ± 2.6	176 ± 3	10.2 ± 2.4	170 ± 5
	15	1	159 ± 34	7.9 ± 3.0	176 ± 3	15.1 ± 2.5	170 ± 3
Right parietal	3	-38	87 ± 57	0.2 ± 0.4	177 ± 1	3.1 ± 1.7	169 ± 7
	6	-24	98 ± 60	1.2 ± 1.3	177 ± 1	6.0 ± 2.2	169 ± 7
	10	-13	117 ± 60	3.5 ± 2.4	177 ± 2	10.0 ± 2.4	169 ± 6
	15	-5	146 ± 44	6.9 ± 3.3	177 ± 2	15.0 ± 2.5	169 ± 5

**Table 5:** Results of experiment on real data.

Subject	Test 1			Test 2 or test 3		
	First sound	Second sound	*P* value	First sound	Second sound	*P* value
S1	3.3 ± 1.7	1.9 ± 1.5	0.009	2.6 ± 1.8	1.2 ± 1.8	0.011
S2	3.0 ± 1.7	1.8 ± 1.4	0.009	2.5 ± 1.8	1.0 ± 1.1	0.010
S3	3.1 ± 1.4	1.7 ± 1.5	0.008	2.9 ± 1.7	1.0 ± 1.0	0.008
S4	3.1 ± 1.4	1.8 ± 1.5	0.012	2.9 ± 1.5	1.2 ± 1.0	0.014
S5	3.0 ± 1.5	1.7 ± 1.1	0.013	2.5 ± 1.7	0.8 ± 0.9	0.009
S6	3.3 ± 1.9	1.9 ± 1.5	0.006	2.4 ± 1.3	0.7 ± 1.0	0.011
S7	2.9 ± 1.5	1.9 ± 1.3	0.017	2.6 ± 1.8	0.6 ± 0.8	0.009
S8	3.0 ± 1.8	1.8 ± 1.6	0.011	2.4 ± 1.7	0.5 ± 0.9	0.009

## Data Availability

The datasets used during the current study are available from the corresponding author on reasonable request.
